The article "Dynamic performances of a bird-like flapping wing robot under randomly uncertain disturbances" was retracted in 2024. Reasons: duplicate publication; overlap with earlier publications; compromised peer review; unreliable results or conclusions.

# Dynamic performances of a bird-like flapping wing robot under randomly uncertain disturbances

**DOI:** 10.1371/journal.pone.0232202

**Published:** 2020-05-05

**Authors:** Changtao Ding

**Affiliations:** Zhejiang Industry Polytechnic College, Shaoxing, Zhejiang Province, China; University College London, UNITED KINGDOM

## Abstract

The nonlinear dynamics of a bird-like flapping wing robot under randomly uncertain disturbances was studied in this study. The bird-like flapping wing robot was first simplified into a two-rod model with a spring connection. Then, the dynamic model of the robot under randomly uncertain disturbances was established according to the principle of moment equilibrium, and the disturbances were modeled in the form of bounded noise. Next, the energy model of the robot was established. Finally, numerical simulations and experiments were carried out based on the above models. The results show that the robot is more likely to deviate from its normal trajectory when the randomly uncertain disturbances are applied in a chaotic state than in a periodic state. With the increase of the spring stiffness under the randomly uncertain disturbances, the robot has a stronger ability to reject the disturbances. The mass center of the robot is vital to realize stable flights. The greater the amplitude of randomly uncertain disturbances, the more likely it is for the robot to be in a divergent state.

## 1. Introduction

In real flights of a bird-like flapping wing robot, the environment is usually not ideal, and there are inevitably randomly uncertain disturbances [1]. The sources of the randomly uncertain disturbances are mainly from the following: (1) Randomly uncertain changes of external loads, such as unexpected slight wind, breeze, strong wind, rainy or snowy weather and sandstorms; (2) Randomly uncertain disturbances generated from the driver, such as vibration of the motor; (3) Friction in the transmission system; (4) Interference from electromagnetic signals [2, 3]. These randomly uncertain disturbances exist commonly in the robot flights and have an important influence on the robot’s dynamics. Thus only in-depth research can ensure the stability of a bird-like flapping wing robot in real flights.

Researchers have extensively studied randomly uncertain disturbances in recent decades. For example, Gaussian white noise was used to model the randomly uncertain disturbances in [4]. X. Leng et al. calculated the randomly uncertain disturbance samples using the power spectral method and researched rotor bifurcation and chaos under the disturbances [5]. White noise and Brownian motion were used to model the randomly uncertain disturbances in [6]. D. D. D. Souza et al studied the randomly uncertain disturbances by characterizing unwanted terms in the Hamiltonians [7]. A linear time invariant system was also used to generate the first-order Markov colored noise to model the small random disturbances in [8]. C. G. Higuera-Chan et al. described the random disturbances with stochastic difference equations, and assumed the disturbances were observable, independent, and uniformly distributed with a density ρ [9]. The randomly uncertain disturbances were regarded as bounded noise processes that were imposed on a system when exploring noise-induced complicated dynamics [10]. Y. Zhuang et al. described the random disturbances by a 3D laser-based measurement and a novel place recognition method [11]. From the above studies, it can be obtained that the randomly uncertain disturbances have been described by different mathematical models.

The article "Dynamic performances of a bird-like flapping wing robot under randomly uncertain disturbances" was retracted in 2024. Reasons: duplicate publication; overlap with earlier publications; compromised peer review; unreliable results or conclusions.

Some dynamic models of flapping wing robots have been established by many researchers in recent decades. Y. Huang et al. simplified a flapping wing robot into two rigid wings connected by a spring, ignored aerodynamic forces and derived the dynamic model based on the balance of linear and angular momenta [12, 13]. C. Bose et al. considered the structural model of a flapping flight as a linkage system, and established the dynamic model in the form of a Duffing oscillator, and used the lumped vortex method to calculate the aerodynamic force of the robot [14]. J. Pohly et al. described the dynamic model of a flapping robot with the Navier-Stokes equation, and obtained the accuracy of a quasi-steady flapping model by analyzing the aerodynamic responses of the robot [15]. In [16], the dynamic model of a flapping wing robot was presented with governing equations and boundary conditions, an energy-based barrier Lyapunov function was used to obtain the robot stability. The efficient and comprehensive dynamic model of a flapping robot was presented with the bond graph method, which can clearly obtain power flows [17]. Some complex interactions were taken into account, S. H. Pourtakdoust et al. used the Euler-Bernoulli torsion beam and the quasi steady aerodynamics to establish the aeroelastic model of a flexible flapping robot [18].

Many researchers have studied robot dynamics under randomly uncertain disturbances. A robot dynamic model was established using the Lagrange-Euler equations, and robot dynamics was established under randomly uncertain disturbances [19]. Bounded noise was used to describe randomly uncertain disturbances, and the dynamics of a bipedal robot was studied in [20]. N. E. Khazen et al. studied the balance of humanoid robots under randomly uncertain disturbances based on the robot dynamics [21]. C. Zaoui et al. established the dynamic model under uncertain disturbances, and identified the robot’s upper part can reject large disturbances based on interactions between dynamic motions and balancing masses [22]. The dynamic results showed that a robot’s disturbance rejection ability can be improved with hip springs [23]. Despite the above studies, there are few studies devoted to model dynamics of a bird-like flapping wing robot under randomly uncertain disturbances.

The article "Dynamic performances of a bird-like flapping wing robot under randomly uncertain disturbances" was retracted in 2024. Reasons: duplicate publication; overlap with earlier publications; compromised peer review; unreliable results or conclusions.

Researchers have employed some methods to analyze dynamic performances of the robot, e.g., the phase diagram method, the Poincaré mapping method. L. Sentis et al. described phase diagrams of the robot CoM (center of mass) with the perturbation theory, the multi-step phase diagrams showed that the robot can walk successfully in rough terrains [24]. In [25], the stability of a passive dynamic walking robot was described by a hybrid Poincaré map, the results showed the stability only depends upon the impact instant. In [26], the Lyapunov’s method was used to analyze the stability of three-DOF (degree of freedom) robots. T. Hase et al. obtained the energy-efficient of a full-actuated robot based on the optimal trajectory planning method, and evaluated the dynamic performances of the robot with the energy-efficiency [27]. T. Fujikawa et al. investigated the dynamic performances of a small flapping robot by analyzing its motion based on the computational models, and clarified the effectiveness of the methodology by experiment results [28,29].

The dynamic performances of a bird-like flapping wing robot under randomly uncertain disturbances were studied in this study. The Sections are arranged as follows: the simplified physical model is first established based on a real bird-like flapping wing robot in Section 2. In Section 3 the dynamic model of the robot is established under randomly uncertain disturbances; both the mathematical model for the randomly uncertain disturbances and the energy model are provided in this Section. Section 4 conducts the dynamic simulations and experiments under randomly uncertain disturbances. Section 5 gives the conclusions and discussion. This study provides an important theoretical basis for the stable flights of a bird-like flapping wing robot in complex environments.

## 2. The simplified physical model of a bird-like flapping wing robot

The bird-like flapping wing robot is shown in Fig 1A. The robot consists of two wings, a torso, and a tail. The airfoil of the robot in Fig 1A is a flat plate. Based on previous researches in the reference [30], the robot can fly in an ideal environment. As shown in Fig 1B, the physical model of the robot can be simplified into two rods with mass *m* and length *l*, ignoring the trunk and tail [11]. Here, the stiffness of the spring that connects the rods is *k*, the randomly uncertain disturbance is *M*, the angle between the swinging rod and the central axis is *α*, the remaining angle between the rod and the central axis is *α*_0_, the angle between the central axis and the vertical line is *θ*, and the acceleration of gravity is *g*.

The article "Dynamic performances of a bird-like flapping wing robot under randomly uncertain disturbances" was retracted in 2024. Reasons: duplicate publication; overlap with earlier publications; compromised peer review; unreliable results or conclusions.

**Fig 1:** The bird-like flapping wing robot and its simplified physical model.

## 3. The robot dynamic model under randomly uncertain disturbances

With only gravity and randomly uncertain disturbances considered, a dynamic model for the bird-like flapping wing robot in Fig 1B is established based on the principle of moment equilibrium, which is shown in Eq (1) [11].

$$\{\begin{array}{l} \frac{2}{3}ml^{2}\ddot{\theta }=-mgl\text{cos}\alpha \text{sin}\theta -M_{1}\\ \frac{2}{3}ml^{2}\ddot{\alpha }=-mgl\text{sin}\alpha \text{cos}\theta -4k(\alpha -\alpha_{0})-M_{2} \end{array}$$ (1)

Where *θ* represents the body dynamics, *α* represents the flapping dynamics. Eq (1) can be rewritten into Eq (2) for normalization:

$$\{\begin{array}{l} \frac{2}{3}ml^{2}\frac{d^{2}\theta }{dt^{2}}=-mgl\text{cos}\alpha \text{sin}\theta -M_{1}\\ \frac{2}{3}ml^{2}\frac{d^{2}\alpha }{dt^{2}}=-mgl\text{sin}\alpha \text{cos}\theta -4k(\alpha -\alpha_{0})-M_{2} \end{array}$$ (2)

Let $t=\tilde{t}/\sqrt{\frac{2l}{3g}}$, $k=mgl\tilde{k}/4$, $M_{1}={\tilde{M}}_{1}mgl$, $M_{2}={\tilde{M}}_{2}mgl$, then,

$$\{\begin{array}{l} \frac{2}{3}ml^{2}\frac{d^{2}\theta }{d{\tilde{t}}^{2}}\frac{3g}{2l}=-mgl\text{cos}\alpha \text{sin}\theta -{\tilde{M}}_{1}mgl\\ \frac{2}{3}ml^{2}\frac{d^{2}\alpha }{d{\tilde{t}}^{2}}\frac{3g}{2l}=-mgl\text{sin}\alpha \text{cos}\theta -4\frac{mgl\tilde{k}}{4}(\alpha -\alpha_{0})-{\tilde{M}}_{2}mgl \end{array}$$ (3)

After simplification and normalization, then,

$$\{\begin{array}{l} \frac{d^{2}\theta }{d{\tilde{t}}^{2}}=-\text{cos}\alpha \text{sin}\theta -{\tilde{M}}_{1}\\ \frac{d^{2}\alpha }{d{\tilde{t}}^{2}}=-\text{sin}\alpha \text{cos}\theta -\tilde{k}(\alpha -\alpha_{0})-{\tilde{M}}_{2} \end{array}$$ (4)

That is

$$\{\begin{array}{l} \ddot{\theta }=-\text{cos}\alpha \text{sin}\theta -M_{1}\\ \ddot{\alpha }=-\text{sin}\alpha \text{cos}\theta -k(\alpha -\alpha_{0})-M_{2} \end{array}$$ (5)

The randomly uncertain disturbances *M*_*i*_ (*i* = 1, 2) generate independently and can be expressed in the form of bounded noise [10, 31, 32], which is shown in Eq (6):

$$M_{i}=A_{i}\text{sin}[\omega_{i}t+\sigma_{i}B_{i}(t)+\gamma_{i}]\;(i=1,2)$$ (6)

where *A*_*i*_ and *ω*_*i*_ are the amplitude and frequency of the randomly uncertain disturbances, respectively, *σ*_*i*_ is a positive constant, *B*_*i*_*(t)* is the unit Wiener process, and *γ*_*i*_ follows a uniform distribution within [0, 2π].

The article "Dynamic performances of a bird-like flapping wing robot under randomly uncertain disturbances" was retracted in 2024. Reasons: duplicate publication; overlap with earlier publications; compromised peer review; unreliable results or conclusions.

Energy *E* can be expressed by Eq (7):

$$E=\frac{1}{2}\left({\dot{\alpha }}^{2}+{\dot{\theta }}^{2}\right)-\text{cos}\alpha \text{cos}\theta +\frac{1}{2}k{\left(\alpha -\alpha_{0}\right)}^{2}-\frac{A_{1}\text{cos}[\omega_{1}t+\sigma_{1}B_{1}(t)+\gamma_{1}]}{\omega_{1}+\sigma_{1}{B^{\prime }}_{1}(t)}-\frac{A_{2}\text{cos}[\omega_{2}t+\sigma_{2}B_{2}(t)+\gamma_{2}]}{\omega_{2}+\sigma_{2}{B^{\prime }}_{2}(t)}$$ (7)

## 4. Simulations and experiments

The dynamic simulations of the robot in an ideal environment were first performed in this section. Then randomly uncertain disturbances were added to study the dynamics in periodic and chaotic states, followed by the dynamic simulations of the robot with different spring stiffnesses under randomly uncertain disturbances. Finally, the dynamic performances of the robot were obtained under randomly uncertain disturbances with different amplitudes.

### 4.1 Dynamic simulations under randomly uncertain disturbances in periodic and chaotic states

In order to integrate over the second order dynamic model shown in Eq (5), let $\dot{\theta }=u_{\theta }$ and $\dot{\alpha }=u_{\alpha }$, then the first order dynamic model is obtained, as shown in Eq (8):

$$\{\begin{array}{l} \dot{\theta }=u_{\theta }\\ \dot{\alpha }=u_{\alpha }\\ {\dot{u}}_{\theta }=-\text{cos}\alpha \text{sin}\theta -M_{1}\\ {\dot{u}}_{\alpha }=-\text{sin}\alpha \text{cos}\theta -k(\alpha -\alpha_{0})-M_{2} \end{array}$$ (8)

Let k = 32, $\alpha_{0}=\frac{\pi }{4}$, and an initial state of $x_{0}=\left[\theta ,\alpha ,\dot{\theta },\dot{\alpha }\right]=\left[\pi /3,\pi /6,0,0\right]$. The simulation results of the periodic dynamics in an ideal environment are shown in Fig 2A and 2B. Then let *k* = 8, $\alpha_{0}=\frac{\pi }{4}$, and an initial state of $x_{0}=\left[\theta ,\alpha ,\dot{\theta },\dot{\alpha }\right]=\left[\pi /2,\pi /4,1.1521,0\right]$. The simulation results of the chaotic dynamics in an ideal environment are shown in Fig 2C and 2D.

**Fig 2:** The dynamic simulations of the bird-like flapping wing robot under an ideal environment.

The simulation results shown in Fig 2 are consistent with the reference [11]. In the following, the amplitudes of randomly uncertain disturbances were set as *A*_1_ = 0.1 and *A*_2_ = 0.1, and the other parameters were the same as that in Fig 2. The dynamic simulations are shown in Fig 3.

**Fig 3:** The dynamic simulations with the parameters in the periodic or chaotic state under randomly uncertain disturbances with the amplitude *A*_1_ = 0.1 and *A*_2_ = 0.1. (a) and (b): phase diagram with the parameters in the periodic state; (c)–(f): dynamic responses with the parameters in the chaotic state. The red dot indicates the equilibrium point.

The article "Dynamic performances of a bird-like flapping wing robot under randomly uncertain disturbances" was retracted in 2024. Reasons: duplicate publication; overlap with earlier publications; compromised peer review; unreliable results or conclusions.

From Fig 3A and 3B, it can be obtained that the equilibrium point locates at the center of the phase diagram, which is similar to Fig 2A and 2B. The $\theta -\dot{\theta }$ curves in Fig 3A do not overlap completely but show a small range of fluctuation. However, no divergent state appears at the end, which indicates that the randomly uncertain disturbances have affected $\theta -\dot{\theta }$ somewhat in the periodic state. The curves in Fig 3B are more concentrated than those in Fig 3A, which indicates the influence of the randomly uncertain disturbances is less on $\alpha -\dot{\alpha }$ and more on $\theta -\dot{\theta }$.

The randomly uncertain disturbances with the amplitudes *A*_1_ = 0.1 and *A*_2_ = 0.1 were added in the chaotic state, and the dynamic simulations of the robot are shown in Fig 3C–3F. The fluctuation range of $\theta -\dot{\theta }$ in Fig 3C is large under the randomly uncertain disturbances. A non-closed curve appears in Fig 3C, which indicates that the robot appears a divergent dynamic state. The curves in Fig 3D are tangled, which appears to be a chaotic state. Fig 3E clearly shows that there are some fluctuations in each period. In the last period, the value of *θ* decreases gradually and eventually fails to return to the normal orbits. The curves in Fig 3F are not smooth and exhibit relatively fast fluctuations, but there is no divergent state, which indicates that the influence of the randomly uncertain disturbances is smaller on $\alpha -\dot{\alpha }$ than on $\theta -\dot{\theta }$. By comparing Fig 3A–3B with Fig 3C–3F, it can be obtained that the robot stability is higher in the periodic state than that in the chaotic state under the randomly uncertain disturbances.

### 4.2 Dynamic simulations with different spring stiffnesses under randomly uncertain disturbances

The effect of spring stiffness *k* on the robot dynamics under randomly uncertain disturbances was investigated in this section. Let *θ* = 0, the energy *E* = 3, the spring stiffness *k* = 1, 10, 20, and all other parameters were the same as those in Fig 3A–3B. The dynamic simulations of the robot with the above parameters are shown in Fig 4.

**Fig 4:** The dynamic simulations of the robot with different spring stiffnesses under the randomly uncertain disturbances. (a) and (b): the spring stiffness *k* = 1; (c) and (d): the spring stiffness *k* = 10; (e) and (f): the spring stiffness *k* = 20. Where (b), (d), and (f) are obtained by projecting the mapping points in (a), (c), and (e) onto the plane in the energy sphere.

The article "Dynamic performances of a bird-like flapping wing robot under randomly uncertain disturbances" was retracted in 2024. Reasons: duplicate publication; overlap with earlier publications; compromised peer review; unreliable results or conclusions.

When the spring stiffness *k* = 1, Fig 4A shows that the Poincaré mapping points are randomly distributed on the outer surface of the energy sphere. There are fewer Poincaré mapping points near the red line. In Fig 4B, the Poincaré mapping points are randomly distributed, which indicates that the robot dynamics is irregular. The interval of the swing angle in Fig 4B is [–2, 3].

When spring stiffness *k* = 10, the Poincaré mapping points in Fig 4C are no longer randomly distributed on the surface of the energy sphere. Instead, the mapping points form a number of rings wrapped around the outer surface of the energy sphere. The Poincaré mapping points in Fig 4D mainly concentrate in two regions: a small elliptical ring inside and a large elliptical ring outside. The interval of the swing angle in Fig 4D is [-0.3, 1.8], which is smaller than that in Fig 4B.

When the spring stiffness *k* = 20, Fig 4E and 4F show that the Poincaré mapping points are not broadly distributed over the surface of the energy sphere, but are concentrated in six circles distributed on the outer surface of the energy sphere. It indicates that the randomly uncertain disturbances have less influence on the flapping wing robot, and the robot has a good stability. The interval of the swing angle in Fig 4F is slightly smaller than that in 4(d). In summary, as the spring stiffness increases, the movements of the robot becomes more stable, and the swing angle becomes smaller.

### 4.3 Dynamic simulations under randomly uncertain disturbances with different amplitudes

To study the influence of different disturbance amplitudes on the robot dynamics, the amplitudes were separately set as *A*_*i*_ = 0.05, 0.5, 5, 20 (i = 1, 2). The other parameters remained the same as those in Fig 3A and 3B. The above randomly uncertain disturbances were added to the dynamic system according to Eq (5), and the simulation results are shown in Fig 5.

**Fig 5:** The dynamic simulations under the randomly uncertain disturbances with different amplitudes. (a) and (b): the amplitude of the disturbances is *A*_*i*_ = 0.05 (*i* = 1, 2); (c) and (d): the amplitude of the disturbances is *A*_*i*_ = 0.5 (*i* = 1, 2); (e) and (f): the amplitude of the disturbances is *A*_*i*_ = 5 (*i* = 1, 2); (g)-(j): the amplitude of the disturbances is *A*_*i*_ = 20(*i* = 1, 2).

Fig 5A and 5B are the phase diagrams when imposing the randomly uncertain disturbances with the amplitude *A*_*i*_ = 0.05 (*i* = 1, 2). From Fig 5A and 5B, the motion of the robot in each period is approximately the same, which indicates that the robot has nearly convergent performances under the above disturbances.

The article "Dynamic performances of a bird-like flapping wing robot under randomly uncertain disturbances" was retracted in 2024. Reasons: duplicate publication; overlap with earlier publications; compromised peer review; unreliable results or conclusions.

From Fig 5C–5F, it can be obtained that as the amplitude of the randomly uncertain disturbances increases, the robot is more likely to deviate from the equilibrium state. Specifically, the degree of fluctuation in Fig 5C is between that in 5(a) and 5(e). When the disturbance amplitude was set as *A*_*i*_ = 5 (*i* = 1, 2), the trajectory of $\theta -\dot{\theta }$ in Fig 5E–5F is different in each period, and $\alpha -\dot{\alpha }$ shows a large range of fluctuation. By comparing Fig 5C–5F, it can be obtained that the fluctuation of $\theta -\dot{\theta }$ is greater than that of $\alpha -\dot{\alpha }$ under the randomly uncertain disturbances, which indicates the mass center of the robot should be first kept stable for flying stably.

From Fig 5G–5j, it can be obtained that the robot seriously deviates from the normal trajectory when the disturbance amplitude was set as *A*_*i*_ = 20 (*i* = 1, 2). Fig 5G shows there is a non-closed curve with large differences in each period. There is also a large fluctuation but no divergent curve in Fig 5H, which indicates that the disturbances have some influences on $\alpha -\dot{\alpha }$. In Fig 5I, the fluctuation of curve *θ* − *t* increases gradually, and it finally fails to return to the normal orbit. In summary, as the amplitude of the randomly uncertain disturbances increases, the fluctuation of the robot dynamic response becomes larger, and the robot is more likely to deviate from its normal orbit.

### 4.4 Experiments

During the flights of a bird-like flapping wing robot, the wind speeds applied on the robot are usually randomly uncertain [1, 33]. The varying wind speed will lead to some randomly uncertain disturbances. Here, flight experiments of the bird-like flapping wing robot were carried out under different wind speeds. Both the robot shown in Fig 1A and the anemometer shown in Fig 6 were used in the experiments.

**Fig 6:** An anemometer used in the experiments.

The bird-like flapping wing robot separately flied under the maximum wind speed *v*_1_ = 0.5(km/h), *v*_2_ = 4.5(km/h) and *v*_3_ = 9.6(km/h), and its flight experiments are shown in Fig 7A–7C respectively.

**Fig 7:** The flight experiments of the robot under different wind speeds, where (a): under the maximum wind speed *v*_1_ = 0.5(km/h), (b): under the maximum wind speed *v*_2_ = 4.5(km/h), and (c): under the maximum wind speed *v*_3_ = 9.6(km/h).

It can be obtained from Fig 7A that the bird-like flapping wing robot can stably fly under the maximum wind speed *v*_1_ = 0.5(km/h), as the randomly uncertain disturbances have weak influence on the robot dynamics. The maximum wind speed in Fig 7B is *v*_2_ = 4.5(km/h), which causes a lot randomly uncertain disturbances. Under this environment, though the robot still flies in the sky, it has some unstable states. In Fig 7C, the robot can not fly normally and falls on the ground, due to the large randomly uncertain disturbances caused by the fastest wind speed *v*_3_ = 9.6(km/h).

The article "Dynamic performances of a bird-like flapping wing robot under randomly uncertain disturbances" was retracted in 2024. Reasons: duplicate publication; overlap with earlier publications; compromised peer review; unreliable results or conclusions.

## 5. Conclusions and discussion

### 5.1 Conclusions

The dynamic performances of the bird-like flapping wing robot under randomly uncertain disturbances were studied in this study. The robot was first simplified into the spring-connected two-rod model, and then the dynamic model was established based on the principle of moment equilibrium. Then the randomly uncertain disturbances were modeled mathematically in the form of bounded noise, and the energy model was also established. Finally, some numerical simulations and experiments of the robot were conducted based on the above models. The results show that the randomly uncertain disturbances have a greater influence on the robot in a chaotic state than in a periodic state. As the spring stiffness increases, the stability of the robot becomes stronger. The mass center is a key factor to ensure fly stably. The greater the amplitude of the randomly uncertain disturbances, the more likely the robot appears in a divergent state.

### 5.2 Discussion

During flights of a bird-like flapping wing robot, there are inevitably some randomly uncertain disturbances from internal friction or weather. These disturbances will prevent the robot from flying normally. Therefore, it is vital to investigate the robot dynamic performances under the randomly uncertain disturbances to ensure stable flights.

The dynamic performances of the robot have been studied in this study. Some measures are concluded to improve the robot stability under randomly uncertain disturbances. To begin with, the parameters in the periodic state (*k* = 32, $\alpha_{0}=\frac{\pi }{4}$ and $x_{0}=\left[\theta ,\alpha ,\dot{\theta },\dot{\alpha }\right]=\left[\pi /3,\pi /6,0,0\right]$) instead that in the chaotic state (*k* = 8, $\alpha_{0}=\frac{\pi }{4}$ and $x_{0}=\left[\theta ,\alpha ,\dot{\theta },\dot{\alpha }\right]=\left[\pi /2,\pi /4,1.1521,0\right]$) should be used during the design and debugging of the robot. Furthermore, it is increasing the spring stiffness (from *k* = 1, then *k* = 10, to *k* = 20) that can effectively improve the anti-disturbance performances of the robot. In the following, the mass center should be given priority to keep stable in the robot flights, as $\theta -\dot{\theta }$ is more easy to fluctuate than $\alpha -\dot{\alpha }$. Finally, the amplitude of randomly uncertain disturbances should be reduced during the robot flights, as the disturbances with the amplitude *A*_*i*_ = 20 (*i* = 1, 2) have a larger effect on the flight stability than that with the amplitude *A*_*i*_ = 5 (*i* = 1, 2), and the flight stability of the robot is the strongest under the disturbances with the amplitude *A_i_* = 0.5 (*i* = 1, 2).

The article "Dynamic performances of a bird-like flapping wing robot under randomly uncertain disturbances" was retracted in 2024. Reasons: duplicate publication; overlap with earlier publications; compromised peer review; unreliable results or conclusions.

In this study, the dynamic model of the robot was established by referring to the reference [11], and then the dynamic performances of the robot in the ideal situation were obtained. The simulation results are consistent with those in the reference [11], which proves the feasibility of this study. In the references [14,24,34,35], the dynamic performances of the flapping wing robot were also studied based on different dynamic models. From the results comparison in the references [11,14,24,34,35], the dynamic performances of the robot are different when different models are established. Even the same model but different parameters are used, different dynamic performances will be obtained. Therefore, it is vital to establish a corresponding dynamic model according to the robot prototype.

In this study, the mathematical model of randomly uncertain disturbances was established based on the bounded noise method, which has been widely used in the previous researches [10,20,31,32,36–40], and its effectiveness has been effectively proved. Based on the above studies, the dynamic model of the robot under the disturbances was established for studying the dynamic performances of the robot. Specially, I have tried to establish the dynamic model of the robot under randomly uncertain disturbances by using the Reynolds-averaged Navier-Stokes (RANS) equation [41–43]. However, it is difficult to obtain simulation results as the calculation amount is very large. Therefore, the real robot was simplified into a two-rod model, and its flight condition was also simplified, which makes the work feasible.

Based on the above models, some conclusions were obtained by carrying out the simulations and experiments. Some useful suggestions on improving the robot stability were got to guide the design and debugging of the robot. For example, periodic motion parameters should be used, the spring stiffness should be increased if anti-disturbance performances of the robot are weak, some measures should be taken to reduce the shaking of the mass center and the disturbance amplitude. As far as I know, these suggestions have rarely studied [44–46]. Though the above conclusions have been obtained, the following aspects should be further studied in the future: (1) A complex dynamic model should be established to approach the real robot under randomly uncertain disturbances, and a method should be proposed to solve the contradiction between the model complexity and the calculation feasibility; (2) Some quantitative conclusions, e.g., the influence mechanism curves of the disturbances on the robot performances, should be further studied; (3) Some other experiments under randomly uncertain disturbances, e.g., wind tunnel experiments, vibration and friction experiments, should be carried out in the future.

The article "Dynamic performances of a bird-like flapping wing robot under randomly uncertain disturbances" was retracted in 2024. Reasons: duplicate publication; overlap with earlier publications; compromised peer review; unreliable results or conclusions.

## Supporting information

S1 File (RAR)
